The article "Diagnosis of Interventional Transvaginal Maternal Diseases Based on Color Doppler Ultrasound" was retracted in 2023. Reasons: signs of a paper mill; suspected computer-generated content; unreliable results or conclusions; lack of ethics approval or compliance.

# Diagnosis of Interventional Transvaginal Maternal Diseases Based on Color Doppler Ultrasound

**DOI:** 10.1155/2021/5517785

**Published:** 2021-04-01

**Authors:** Canliang Wen, Lan Huang, Hongye Jiang

**Affiliations:** ^1^Department of Obstetrics and Gynecology, Guangzhou Women and Children's Medical Center, Guangzhou, Guangdong 510623, China; ^2^Department of Ultrasound, Guangzhou Women and Children's Medical Center, Guangzhou, Guangdong 510623, China; ^3^Department of Obstetrics and Gynecology, The First Affiliated Hospital, Sun Yat-sen University, Guangzhou, Guangdong 510080, China

## Abstract

In recent years, with the development of color Doppler ultrasound technology in obstetrics, this noninvasive, direct, convenient, and sensitive inspection method has become one of the best methods to observe the fetal circulation in the uterus. This paper discusses the clinical value of using transvaginal color Doppler ultrasound in the differential diagnosis of ovarian corpus luteum disease and ectopic pregnancy disease. This paper selects 100 cases of ectopic pregnancy and 100 cases of pregnant corpus luteum as the experimental research objects. Clinical analysis of transvaginal color Doppler ultrasonography was performed on all patients. In the process of measuring the patient's ectopic pregnancy, the size of the patient's adnexal mass is mainly measured, and the blood flow spectrum is measured. The clinical choice of transvaginal color Doppler ultrasound method to distinguish ectopic pregnancy disease and corpus luteum pregnancy disease can play a significant value. It can be effectively diagnosed according to the type of disease, then effective methods can be studied for clinical treatment, the quality of life of patients with the two diseases can be significantly improved, and the clinical application value of color Doppler ultrasound can be improved.

## 1. Introduction

In recent years, with the development of color Doppler ultrasound technology in obstetrics, this noninvasive, direct, convenient, and sensitive inspection method has become one of the best methods to observe the fetal circulation in the uterus. The application of color Doppler ultrasound technology can not only improve the observation level of morphology but also detect intrauterine blood flow parameters and hemodynamic characteristics, which can help evaluate fetal distress and pregnancy prognosis [1]. In this study, the US GE Voluson E8 color Doppler ultrasound diagnosis system first performed routine ultrasound examinations to understand the general condition of the fetus, such as fetal double parietal diameter, head circumference, abdominal circumference, femur length, ocular bone length, amniotic fluid volume, placental position, placental thickness, and maturity. Ultrasound imaging uses sound waves to produce pictures of the inside of the body. It is used to help diagnose the causes of pain, swelling, and infection in the body's internal organs and to examine a baby in pregnant women and the brain and hips in infants. It is also used to help guide biopsies, diagnose heart conditions, and assess damage after a heart attack. Ultrasound is safe and noninvasive and does not use ionizing radiation. After a series of indicators, the blood flow indexes of the fetus are measured, the above detection values are compared with other hypoxia indicators of the perinatal infant, and the combined detection of blood flow indexes of different organs of the fetus can be used to predict fetal hypoxia and to evaluate the clinical value of perinatal outcomes [2].

Ectopic pregnancy, as a relatively serious obstetric acute abdomen in clinical practice, has shown a gradual increase in incidence in recent years and is also the main cause of death for pregnant women. From a clinical analysis, the corpus luteum of pregnancy is a special type of mass, which is mainly a cystic mass that appears inside the ovaries of the pregnant woman during the early pregnancy. In most cases, the corpus luteum of the ovary of pregnancy will gradually shrink and disappear with the continuous increase of the number of weeks of pregnancy of the pregnant woman [3]. Therefore, the corpus luteum of pregnancy and ectopic pregnancy have a certain crossover phenomenon in two-dimensional sound imaging, color blood flow, and so on, and clinical misdiagnosis is easy to occur. The differential diagnosis of ovarian corpus luteum and ectopic pregnancy by transvaginal color Doppler ultrasound was discussed.

This paper selects patients with ectopic pregnancy and pregnant corpus luteum as the experimental research objects. The first part is the clinical implementation of transvaginal color Doppler ultrasound for all patients and introduces the application of transvaginal color Doppler ultrasound. Subsequently, in the process of measuring the patient's ectopic pregnancy, the size of the patient's adnexal mass is measured, and the blood flow spectrum is measured. In the process of measuring the corpus luteum of pregnancy, the size of the corpus luteum and the blood flow spectrum of the patient are measured. For patients with ectopic pregnancy, the size of the mass is different. Ultrasound examinations were performed on the patients, and the final examination results showed a gestational sac type and heterogeneous echogenic mass. During ectopic pregnancy, the masses are mainly strip-shaped and spot-shaped blood flow, the frequency spectrum is mostly extremely low resistance, and the blood flow comes from outside the ovary. Observation of the types of ultrasound manifestations found that the main manifestations were hypoechoic, thin-walled cysts, and thick-walled double rings. Bright, thick, continuous circular, or semicircular blood flow signals can be seen around the corpus luteum of pregnancy. The frequency spectrum is mostly low resistance and high resistance. The blood flow comes from the ovaries. Finally, it is concluded that the clinical choice of transvaginal color Doppler ultrasound to distinguish ectopic pregnancy disease and corpus luteum pregnancy disease can play a significant role. It can be effectively diagnosed according to the type of disease, and then effective methods are studied for clinical treatment. The quality of life is significantly improved, showing the clinical application value of color Doppler ultrasound.

## 2. Related Work

Three-dimensional color Doppler ultrasound is a three-dimensional dynamic display color Doppler ultrasound diagnostic instrument, with special features such as stereo imaging, image cutting, image rotation, and high plane image analysis. In the ultrasound image, the normal placenta appears as follows: the posterior placenta space is clearly visible. It is composed of three parts: the decidua interface with strong echo, the hypoechoic myometrium, and the echoless posterior placental blood vessel [3].

Depending on the depth and range of the placenta implantation into the myometrium, the prenatal performance of three-dimensional color Doppler ultrasound in the placenta implantation can have different sound and image characteristics. Garmendia et al.'s [4] studies have shown that the three-dimensional color Doppler ultrasound images of placenta accreta have the following characteristics: the distribution of blood vessels around the placenta is abnormal, manifested by increased, thickened, and irregular arrangements of blood vessels; the area is accompanied by pulse perfusion or turbulence; that is, blood flow in the placental cavity is formed. Liu et al. [5] analyzed 8 patients with lacunar blood flow on ultrasound and confirmed that 7 cases were placenta accreta, which may be related to abnormal microvascular dynamics in the villous space. The formation of lacunar blood flow may be due to the low decidual response of this type of placenta, which causes extravillous trophoblast cells to invade the deep muscle layer. At this time, the blood vessels originally confined to spiral arterioles expand to a larger size. For the arcuate arteries, the high pulse pressure blood flow of the deep arteries formed the lacunar blood flow under ultrasound. However, Puente's study [6] believes that the possible mechanism of placental implant ultrasound performance is as follows: long-term exposure to pulsed blood flow can form a “spout effect.” In this process, tissue infarction, fibrosis, and other pathological changes can cause damage. The degeneration and thinning shown in the ultrasound image are anechoic dark areas of the placenta. On this basis, some studies have put forward the key points for the diagnosis of lacunar blood flow:

1. The width of the echogenic dark area in the placenta due to lacunar blood flow is greater than 1 cm, and its content contains multiple small compartments to form a blood pool.
2. The whole layer from the placental base plate to the villi plate is occupied.
3. After increasing the frame rate, the blood flow will be pulsed or laminar under ultrasound.
4. The boundary between the placenta and the muscle layer and related tissues is not clear.
5. Dilated pulsed blood vessels can be seen in the placenta and nonplacental tissues.

Three-dimensional power Doppler ultrasound (3D-PDU) is a technology that combines three-dimensional ultrasound and power Doppler imaging. It can display the structure and structure of blood vessels in a certain unit volume of the detected tissue. For blood flow, the Doppler energy difference is related to the density of red blood cells, scatterers, and amplitude. Therefore, it can provide the perfusion of blood flow in the tissue [7]. 3D-PDU first appeared in the mid-1990s; mainly, it has the following advantages: it is not affected by the ultrasound incident angle and blood flow velocity and can display low-velocity, low-flow blood flow. When the average blood flow velocity in the perfusion area is 0, its energy integral is not. Compared with three-dimensional color Doppler ultrasound, the three-dimensional energy mode can more intuitively display the three-dimensional distribution of blood vessels under the placenta and can better evaluate the placenta accreta. The scope and quantitative assessment of blood perfusion in target organs or tissues can better guide clinical evaluation and treatment [8]. The reconstruction effect of 3D-PDU three-dimensional vascular space structure is similar to angiography technology, but it is safe and noninvasive; there is no need to take contrast agent, avoiding related risks. It can detect low-velocity blood flow more sensitively, which is suitable for the detection of low-velocity blood flow in the placenta. It can quantitatively analyze the blood flow signals of blood vessels in the region of interest. The data are objective and credible.

The blood vessels in the vascular bed in the placenta are thin and small, the flow rate is very low, and there are many blood vessels perpendicular to the ultrasonic sound velocity, so the three-dimensional color Doppler image cannot be displayed; the most prominent advantage of 3D-PDU is that it can detect more low-speed blood flow without being affected by the incident angle of ultrasound [9]. For example, Hutchinson et al. [10] conducted research on abnormal blood vessel reconstruction and showed that when placenta previa is complicated with placenta accreta, abnormally reconstructed blood vessels between the uterus and placenta can improve the diagnostic rate of placenta accreta.

In recent years, there have been many reports on the application of 3D-PDU technology for prenatal diagnosis of placental implants. Kingdom et al. [11] reported a case of using 3D-PDU to diagnose a placenta accreta at 28 weeks of pregnancy and found that when two-dimensional ultrasound is suspected of having a placenta accreta, the application of 3D-PDU revealed obvious abnormalities between the placenta and its surrounding tissues. The vascular branches of blood flow have irregular and abnormal blood supply in the blood perfusion area. In these areas, high-speed turbulent venous blood flow and prominent low-impedance arterial blood flow in the uterus and bladder area can be easily observed (blood flow) by resistance index (RI). 3D-PDU technology for diagnosing placenta accreta has the following characteristics and advantages [12]. Three-dimensional reconstruction technology is an important auxiliary tool for three-dimensional color power Doppler ultrasound, which can display clear vascular structures and at the same time from different perspectives observe the scanning plane to quantify the abnormal uterine placental blood vessels and predict the degree of invasion of the bladder muscle. Because the incidence and mortality of placental implants are closely related to the degree of bladder invasion, it can be accurately diagnosed before delivery. The degree will help doctors prepare for surgery and manage the perinatal period of patients. “Wall display mode” can cut the area between the bladder and the uterus to form multiple parallel planes, which are very similar to the multiplanar observation of CT, which can accurately assess the position and range of blood vessels invading the myometrium and bladder skin and the depth of invasion. It can accurately and quantitatively evaluate abnormal neovascularization through three-dimensional ultrasonic volume automatic measurement technology. However, at present, there is no uniform standard for evaluating the blood supply of placenta by using 3D-PDU. In order to diagnose placenta accreta more objectively and accurately, multicenter, large-sample clinical research is currently required to obtain normal reference values of placental blood flow of pregnant women in different periods. The diagnosis of maternal diseases is shown in Figure 1.

## 3. Materials and Methods

### 3.1. General Information

From January 2018 to January 2019, 100 patients with ectopic pregnancy and 100 patients with corpus luteum of pregnancy were selected as the research objects of this experiment. There were a total of 200 patients with ectopic pregnancy. The clinical menopause time of the patients was between 35 and 64 days. The age of the patients hovered between 23 and 46 years, with an average age of 29.4 ± 1.2 years. After clinical examination, it was found that the urine *β*-HCG results of 80 patients with ectopic pregnancy were positive, which was finally confirmed as tubal pregnancy. There are a total of 80 patients with corpus luteum during pregnancy. The menopause time of the patients is between 34 and 62 days, and the age of the patients is between 21 and 42 years, with an average age of 30.2 ± 1.1 years. After clinical examination, it was found that 100 cases of pregnant ovarian corpus luteum showed positive urine *β*-HCG, which was finally confirmed to be pregnant ovarian corpus luteum. Observing general data such as the age of patients with ectopic pregnancy and corpus luteum of pregnancy, there is no significant difference (*P* > 0.05).

### 3.2. Method

Transvaginal color Doppler ultrasonography performed clinical diagnosis for all patients. In the process of measuring the patient's ectopic pregnancy, the size of the patient's adnexal mass is mainly measured, and the blood flow spectrum is measured. In the process of measuring the corpus luteum during pregnancy, the size of the corpus luteum and the blood flow spectrum of the patient are measured. In the study, choose to use PHILIPS HD11XE color Doppler ultrasound diagnostic apparatus for diagnosis and analysis, through the patient's vagina for exploration, and control the frequency of the probe between 4 and 8 MHz [12]. In the process of preparing for the implementation of clinical examinations, the main arrangement is for the same clinician to conduct effective examinations. The patient's bladder needs to be effectively emptied, the position of the bladder lithotomy is selected, and the patient's vagina is subjected to ultrasound examination [13]. Secondly, according to the conventional method, check whether there is a gestational sac inside the patient's uterus and observe whether there is a mass in the patient's double appendage area. Third, during the clinical examination, the masses of the two groups of patients were measured reasonably and carefully. Fourth, choose Color Doppler Flow Imaging (CDFI) to carefully observe the blood supply of the two groups of patients, and accurately measure the blood flow parameters of the patients [14]. The transvaginal color Doppler ultrasound detection method is shown in Figure 2.

### 3.3. Judgment Criteria

Color Doppler ultrasound technology can be used to detect the hemodynamics of fetal-related blood vessels and determine the ratio of the end-systolic peak and the end-diastolic peak of the flow velocity (systolic/diastolic, S/D), RI and Pulsatility Index (PI) are used to determine whether the fetus is hypoxic and to predict some possible adverse pregnancy consequences by understanding the blood supply of the fetus in the uterus. The principle is as follows: when the probe of an ultrasound instrument is aimed at the place when selecting the blood vessel (artery) to be detected, the instantaneous Doppler frequency shift between the emitted and reflected waves will be obtained, and the color blood flow spectrogram will be obtained by using the signal processing and imaging technology of the instrument. Its hemodynamics theoretical formula is as follows:

(1) $$\begin{array}{c} \text{SD}=\frac{\text{peak systolic velocity}\left(\text{S}\right)}{\text{end diastolic blood flow velocity}\left(\text{D}\right)},\\ \text{RI}=\text{peak systolic velocity}\left(\text{S}\right)-\frac{\text{end diastolic velocity}\left(\text{D}\right)}{\text{peak systolic velocity}\left(\text{S}\right)},\\ \text{PI}=\text{peak systolic velocity}\left(\text{S}\right)-\frac{\text{end diastolic velocity}\left(\text{D}\right)}{\text{mean velocity}\left(V_{\text{mean}}\right)}. \end{array}$$

The uterine spiral artery, as a branch of the uterine artery (UTA), is the final link of the maternal blood circulation, mainly through the circulation of the placenta to supply the fetus with the nutrients needed during the growth and development process. The changes in various blood flow parameters may indicate the uterus early. According to related literature reports, the higher the circulatory resistance of the posterior spiral artery of the placenta, the worse the prognosis of the fetus. At present, there have been reports in foreign countries using color Doppler ultrasound to detect the hemodynamic indicators of the uterine spiral artery to evaluate the growth status of the fetus in the uterus [15]. The blood flow indicators of blood vessels may reflect changes in arterial dilation and contraction function and changes in the instantaneous resistance of arterial blood flow. By detecting the rate of blood flow, it is possible to reflect the resistance of the placenta and peripheral microcirculation in the case of the fetal umbilical artery (UA), as well as the S/D, IR, and PI values of various resistance indicators. The amount of placental hemoperfusion predicts fetal movement in the womb and the prognosis of the perinatal baby. The spectral Doppler indices measured at the fetal end, the free loop, and the placental end of the umbilical cord are different with the impedance highest at the fetal end. The changes in the indices are likely to be seen at the fetal end first. Ideally, the measurements should be made in the free cord; however, for consistency of recording in cases being followed up, a fixed site would be more appropriate, that is, fetal end, placental end, or intra-abdominal portion. There are also related studies, but reports on combining these two indicators to detect and comprehensively evaluate their predictive value for high-risk pregnancy outcomes are still rare.

The criteria for clinical implementation of extremely low resistance blood flow spectrum judgments are RI below 0.4; for low resistance blood flow spectrum judgment standards, RI is between 0.4 and 0.5; for high resistance blood flow spectrum judgment, the standard is as follows: RI is between 0.51 and 0.99. The color Doppler sonogram of patients with ectopic pregnancy and corpus luteum is shown in Figure 3.

### 3.4. Statistical Methods

CDFI not only has the advantages of real-time, noninvasive, simple, fast, high sensitivity, repeatable inspection, low cost, and so on but also measures various resistance indicators of vascular blood flow, especially for the fetus in the third trimester. The clinical practical value of timely ultrasound detection has been continuously concerned and studied by scholars at home and abroad. As a good method for noninvasive observation of fetal blood circulation in utero, its important value has been universally recognized by sonographers, obstetricians, and gynecologists. As early as 1977, Fitz Gerald used Doppler ultrasound to examine the fetal UA for the first time. Since the blood flow, there have been many related studies and reports at home and abroad [15]. The Doppler blood flow changes of the fetus are often manifested earlier than electronic fetal heart monitoring or biophysical scores. Therefore, color Doppler ultrasound technology can be used to detect fetal blood vessel hemodynamics, determine the ratio of the end-systolic peak of blood flow to the end-diastolic peak, RI, and PI, understand the fetal blood supply, and predict fetal hypoxia and the possible outcome of pregnancy. The overall trend shifted from a single blood vessel and a single indicator to multiple blood vessels and combined detection of multiple indicators. By judging the progress and possible adverse outcomes of high-risk pregnancy, as well as the growth and development of the fetus, it provides a powerful diagnostic basis for clinical termination of abnormal pregnancy, correction of maternal and child abnormalities, and smooth progress of normal pregnancy [16]. The method of using Doppler ultrasound to study the blood circulation status of the fetus at present mainly involves the UA, middle cerebral artery (MCA), venous catheter (DV), renal artery (RA), and abdominal aorta (AA) at home and abroad, and UTA. Currently, UA and UTA hemodynamic testing has been widely used in clinical practice [17]. The diameter of UA is relatively thick and it is the easiest to display, but as a bridge blood vessel between the fetus and the placenta, its blood flow parameters are related to not only the fetus's own condition but also the maternal placenta, so there are certain limitations in predicting the fetus and prognosis; RA diameter is relatively small and easily affected by fetal movement and respiration and is difficult to obtain. However, the fetal kidney is an important organ with rich blood perfusion in the body. RA blood flow parameters can better reflect the fetus's own conditions, and its clinical value has been a large number of scholars at home and abroad. Research has confirmed that the first trimester of pregnancy is due to the obvious decline in MCA color blood flow display due to head-up, and the detection is limited; although the blood flow measurement of the UTA is richer than the blood flow measurement of the uterine placental bed, it can be more conveniently obtained, but the spiral artery is the terminal branch of the UTA, so it can reflect the mother earlier than the UTA and UA [18]. Basic and clinical medicine in the past 20 years has shown that various hemodynamic indicators can provide unique information on the safety of the fetus. Combined testing is more sensitive and reliable than a single indicator. It should be combined with other clinical examinations to make it effective for eugenics and health. Perinatal medicine plays an important role. As we all know, in many clinical testing methods, fetal UA blood flow testing is the most widely used, and the uterine spiral artery is the branch vessel of the UTA, the final link of the maternal blood circulation, mainly through the circulation of the placenta to supply the fetus for growth. The nutrients needed during development and the changes in blood flow parameters may prompt the uterus early. At present, there have been reports in foreign countries using color Doppler ultrasound to detect the hemodynamic indicators of the uterine spiral artery to evaluate the growth status of the fetus in the uterus [19]. There are also related studies in the country, but reports on the combination of these two indicators at the same time and comprehensive evaluation of their predictive value for high-risk pregnancy outcomes are still rare.

The data collected were analyzed using software SPSS Version 17.0 for Windows (SPSS, Chicago, Illinois). The *χ*^2^ test was performed on the spectrum shape and *T*-statistical analysis of the data of patients with ectopic pregnancy and corpus luteum of pregnancy. When *P* < 0.05, there is a significant difference and statistical significance.

## 4. Discussion of Experimental Results

### 4.1. Color Doppler Blood Flow Distribution

For patients with ectopic pregnancy, the size of the mass is different. Ultrasound examinations were performed on the patients, and the final examination results showed gestational sac type and heterogeneous echogenic mass. If the cell is fertilized, the corpus luteum will be affected by the action of HCG, which will continue to grow, continue to grow, and eventually evolve into the pregnant ovarian corpus luteum. Bright, thick, continuous circular, or semicircular blood flow signals can be seen around the corpus luteum of pregnancy. The frequency spectrum is mostly low resistance and high resistance. The flow rate is 18 to 38 cm/s. The blood flow comes from the ovary. During ectopic pregnancy, the mass envelope is formed by decidual cells, muscle fibers, and knot tissue, and the blood supply is poor. Therefore, the blood flow is mainly striped and spotted. The frequency spectrum is mostly extremely low resistance, the flow rate is 8∼25 cm/s, and blood flow comes from outside the ovary. The size of the upper and lower diameters of the corpus luteum during pregnancy is 18.40 ± 2.66 mm; the front and rear diameters are 16.49 ± 2.87 mm; the left and right diameters are 18.07 ± 3.15 mm. Observation of the types of ultrasound findings showed that the main manifestations were hypoechoic, thin-walled cysts, and thick-walled double rings; the clinical choice of transvaginal color Doppler ultrasound to identify ectopic pregnancy disease and luteal disease of pregnancy can play a significant value. The blood flow spectrum shape and blood flow distribution can be seen in Table 1 and Figure 4.

After the female mature follicle ovulates, the follicular wall collapses, and the blood vessels and connective tissue inside the follicular membrane deepen into the granular layer. Due to the series of luteinizing hormones, the volume of the follicular wall cell appears to increase to a certain extent. After continuous action, it will differentiate into endocrine cell clusters rich in blood vessels, which is the clinical corpus luteum. If the egg cell is fertilized, the corpus luteum will be affected by the action of HCG, and it will continue to grow and eventually evolve into the corpus luteum of pregnancy. Bright, thick, continuous circular, or semicircular blood flow signals can be seen around the corpus luteum of pregnancy. The frequency spectrum is mostly low resistance and high resistance. The flow rate is 18 to 38 cm/s. The blood flow comes from the ovary. During ectopic pregnancy, the mass envelope is formed by decidual cells, muscle fibers, and knot tissue. The blood supply is poor, so the blood flow is mainly striped and spotted. The frequency spectrum is mostly very low resistance, the flow rate is 7∼27 cm/s, and blood flow comes from outside the ovary. The clinical analysis statistics of Doppler blood flow spectrum morphology of the two groups of patients are shown in Table 2 and Figure 5.

For patients with ectopic pregnancy and ovarian corpus luteum of pregnancy, the method of “transvaginal color Doppler ultrasound diagnosis” is selected clinically, which can accurately detect and analyze the patient according to the patient's clinical manifestations and clinical indicators and determine the patient's blood flow signal. The blood flow spectrum information is fully collected, and finally, an accurate diagnosis is made for the patient, which provides more references for subsequent clinical treatment and intervention. Compared with general diagnostic methods, transvaginal color Doppler ultrasound diagnosis has the advantages of fast diagnosis, low misdiagnosis rate, and simple operation during the application process. For patients, this diagnostic method has nothing to do with it. Pain reduces the psychological pressure of patients.

### 4.2. The Hemodynamic Indexes in the Normal Pregnancy Group, Ectopic Pregnancy, and Pregnant Corpus Luteum Group

The normal pregnancy group, ectopic pregnancy, and pregnancy corpus luteum group can clearly display MCA and RA. The measured PI, RI, and S/D values are as follows. Comparing the MCA hemodynamic indexes of the ectopic pregnancy group and the normal pregnancy group, the PI, RI, and S/D values of MCA were lower than those of the normal pregnancy group (*P* < 0.01). Comparing the MCA hemodynamic indexes between the ectopic pregnancy group and the pregnant corpus luteum group, the RI and S/D values of MCA were lower than those of the pregnant corpus luteum group (*P* < 0.01), and there was no significant difference in PI value (*P* > 0.05), as shown in Table 3 and Figure 6.

The MCA of the fetus is the blood vessel with the most abundant blood supply to the fetal cerebral hemisphere. Whether the fetal cerebral circulation fluctuates can be clearly shown through it. This study suggests that, compared with normal pregnant fetuses, the fetal MCA RI of the ovarian corpus luteum group are lower than those of the normal pregnancy group, and the difference is statistically significant (*P* < 0.01); compared with normal pregnant fetuses, the fetal MCA RI of the ectopic pregnancy group was lower than the normal pregnancy group, and the difference was statistically significant (*P* < 0.05). In the normal pregnancy, blood flow resistance such as S/D, PI, and RI in the MCA blood flow of the fetus showed a downward trend as the number of weeks of pregnancy increased [14].

Figure 7 shows that, with the continuous development of the embryo and the gradual increase of the brain volume, the blood vessels of the central organs of the fetus have gradually developed more systematically and functioned as the pregnant woman's gestational age continues to grow. The internal blood flow increases, and the amount of oxygen carried by the blood also increases.

After repeating the test several times, compared to the ectopic pregnancy group, the PI of the MCA fetal and the S/D of the luteal fetal group were lower than those of the ectopic pregnancy group, and the difference was statistically significant (*P* < 0.01). In the ectopic pregnancy group, the difference was not statistically significant (*P* > 0.01). This means that when a high-risk pregnancy occurs, resistance to blood flow from the fetal brain is reduced, first ensuring a blood supply to the central organs. When fetal hypertension during pregnancy is in a chronic hypoxic environment, blood circulates through self-compensating physiological regulation of the fetal nerves to ensure blood supply of important central organs such as the brain and heart. It can be redistributed, thickening and dilating the diameter of blood vessels in the central organs of the fetus, thereby reducing the vascular resistance in the central organs and effectively increasing blood flow. At the same time, peripheral blood circulation changes in reverse, blood vessels constrict, and tubes become smaller in diameter. Since then, vascular resistance has increased significantly and blood flow has decreased rapidly, allowing the blood supply to the fetal central organs in intrauterine hypoxia to be maintained.

## 5. Conclusion

In the process of transvaginal ultrasound examination, the probe is close to the cervix and vaginal vault, and the ion uterus and accessories are very close, which reduces the patient's obesity, gas in the intestinal cavity, and other external factors. The high sound image is convenient for early and more accurate inspection. Transvaginal color Doppler ultrasound can not only provide high-resolution, high-definition two-dimensional images but also observe the blood flow changes and spectral characteristics of ectopic pregnancy, which is significantly better than transabdominal ultrasound. It has a high diagnostic accuracy rate, especially for the early diagnosis of ectopic pregnancy with atypical clinical manifestations and cannot be diagnosed by abdominal ultrasound. When an early ectopic pregnancy is suspected, transvaginal ultrasound should be given priority. For patients with ectopic pregnancy and ovarian corpus luteum of pregnancy, transvaginal color Doppler ultrasound diagnosis can be used for differential diagnosis, which can obtain accurate diagnostic results, which has a positive effect on patients and is worthy of clinical application.

## Figures and Tables

**Figure 1:** Diagnosis of maternal diseases.

**Figure 2:** Transvaginal color Doppler ultrasound detection method.

**Figure 3:** Color Doppler sonogram of patients with ectopic pregnancy and corpus luteum.

**Figure 4:** Clinical statistics of patient color Doppler blood flow distribution.

**Figure 5:** Ultrasound imaging of blood flow inside the ovary.

**Figure 6:** The resistance indexes (RI) of the fetal middle cerebral artery (MCA) in the normal pregnancy group.

**Figure 7:** Comparison of the MCA in the normal pregnancy group, ectopic pregnancy, and pregnancy corpus luteum group.

**Table 1:** Clinical statistical analysis of color Doppler blood flow distribution in two groups of patients (cases).

Mass nature	Number of cases	Circular blood flow	Semicircular blood flow	Punctate blood flow	Blood flow comes from inside the ovary	Blood flow comes from outside the ovary
Ectopic pregnancy	100	26	34	40	0	100

Pregnancy corpus luteum	100	62	17	21	100	0

*χ* ^2^	6.348		8.386	10.313	8.946	7.486

*P*	< 0.001		< 0.001	< 0.05	< 0.001	< 0.05

**Table 2:** Clinical analysis statistics of Doppler blood flow spectrum morphology of the two groups of patients (cases).

Mass nature	Number of cases	Very low resistance spectrum	Low resistance spectrum	High resistance spectrum	No diastolic spectrum	Reverse diastolic spectrum
Ectopic pregnancy	100	40	26	14	10	10
Pregnancy corpus luteum	100	0	62	38	0	0
*χ* ^2^	8.347		9.362	10.367	8.953	7.486
*P*	< 0.05		< 0.05	< 0.001	< 0.001	< 0.05

**Table 3:** Comparison of PI, RI, and S/D of fetal MCA in the normal pregnancy group, ectopic pregnancy, and pregnant corpus luteum group (*x* ± *s*).

	Normal pregnancy group (80)	Ectopic pregnancy (100)	Pregnancy corpus luteum group (100)
PI	1.76 ± 0.24	1.21 ± 0.14	0.65 ± 0.05
RI	0.57 ± 0.34	0.53 ± 0.05	4.34 ± 0.32
S/D	1.24 ± 0.14	4.12 ± 0.08	3.48 ± 0.21

## Data Availability

The datasets generated and/or analyzed during the current study are available from the corresponding author upon request.
